# The Anesthetic Effect of Ultrasound-Guided Serratus Anterior Plane Block in Arthroscopic Shoulder Surgery and Its Effect on Postoperative Analgesia

This article has been retracted.

**DOI:** 10.1155/2022/8968805

**Published:** 2022-03-15

**Authors:** Hao Zhu, Chao Zhang, Caoxin Yan

**Affiliations:** ^1^Ultrasound Department of Lanxi People's Hospital, Lanxi 321100, Zhejiang, China; ^2^Ultrasound Department of the Second Affiliated Hospital of Medical College of Zhejiang University, Hangzhou 310000, China; ^3^Department of Ultrasound in Medicine, The Fourth Affiliated Hospital of Zhejiang University School of Medicine, Yiwu, Zhejiang 322000, China

## Abstract

**Objective:**

To investigate the anesthetic effect of anterior serratus muscle plane block under ultrasound guidance in arthroscopic shoulder surgery and its effect on postoperative analgesia.

**Methods:**

A total of 94 patients who received arthroscopic shoulder surgery in our hospital were selected as the research subjects, and they were divided into a control group and a study group according to the random number table method. The control group underwent brachial plexus block under ultrasound guidance, and the study group underwent anterior serratus plane block under ultrasound guidance. The visual analogue score (VAS) of pain at each time point, intraoperative anesthetic dosage, the use of postoperative analgesic, pain mediators and oxidative stress factors before and after surgery, and the occurrence of adverse reactions were compared between the two groups after surgery.

**Results:**

At 6, 12, 48, and 72 h after surgery, there was no obvious difference in the VAS score between the two groups (*P* > 0.05); 24 h after surgery, the VAS score of the study group was significantly lower than that of the control group (*P* < 0.05). The intraoperative dosage of propofol and remifentanil in the study group was significantly lower than that in the control group (*P* < 0.05). The number of effective compressions of analgesic pump and the total amount of sufentanil in the study group were significantly lower than those in the control group within 48 hours after operation, and the time of first compressions of analgesic pump was significantly longer than that in the control group (*P* < 0.05). Before surgery, there were no significant differences in CGRP, NPY, and MDA levels and SOD enzyme activity between the two groups (*P* > 0.05). After surgery, the levels of pain mediators CGRP and NPY in the study group were lower than those in the control group (*P* < 0.05). The level of MDA was lower than that of the control group, and SOD enzyme activity was higher than that of the control group (*P* < 0.05). There was no significant difference in the incidence of adverse reactions between the two groups (*P* > 0.05).

**Conclusion:**

Ultrasound-guided anterior serratus plane block for arthroscopic shoulder surgery has a good anesthesia effect and long action time. It can significantly reduce the dosage of opioids, enhance the postoperative analgesic effect, effectively inhibit postoperative pain and oxidative stress reaction, and has good safety.

## 1. Introduction

Arthroscopic shoulder surgery has been widely used in the treatment of shoulder diseases (such as rotator cuff tear) due to its advantages of minimal invasiveness and safety [1, 2]. However, patients often have severe pain after surgery, which is not conducive to rapid recovery [3, 4]. Therefore, it is very important to find an effective way of anesthesia and analgesia. Brachial plexus nerve block is considered to be the gold standard for analgesia in arthroscopic shoulder surgery and has a good analgesic effect. However, since the posterolateral branch of the shoulder also receives sensory branches from the thoracic nerve, the arthroscopic port entrance in this area may cause pain in the patient during arthroscopic surgery [5, 6]. Relevant studies have found that ultrasound-guided anterior saw muscle plane block can achieve good anterior lateral chest wall analgesia by injecting local anesthetics into the anterior saw muscle and blocking the lateral cutaneous branch of intercostal nerve, which has a significant analgesic effect on patients undergoing thoracoscopy [7, 8]. However, its clinical effect in arthroscopic shoulder surgery is not very clear at present. This study will investigate the anesthetic effect of ultrasound-guided serratus anterior plane block in arthroscopic shoulder surgery and its effect on postoperative analgesia. The results are as follows.

## 2. Material and Methods

### 2.1. General Data

A total of 94 patients who underwent arthroscopic shoulder surgery in our hospital from February 2018 to March 2020 were divided into a control group (47 cases) and a study group (47 cases) according to the random number table method. This study has been approved by the hospital's ethics committee. Inclusion criteria were (1) patients who were diagnosed as rotator cuff tear before surgery and underwent arthroscopic rotator cuff suture surgery; (2) American Society of Anesthesiologists Classification (ASA) [9] Grade I∼II; and (3) those who have given informed consent to the study and signed the informed consent. Exclusion criteria were (1) patients with contraindications/anesthesia; (2) chronic pain or mental illness; and (3) patients with diseases of heart, liver, and other important organs. There was no statistical difference in general data between the two groups (both *P* > 0.05), which are comparable, as shown in Table 1.

### 2.2. Methods

All patients were routinely abstained from drinking and fasting before surgery, and establishing a venous vascular pathway monitored their blood pressure, blood oxygen saturation, heart rate, and other related indicators. All of them received tracheal intubation and general anesthesia. Anesthesia induction was performed using propofol 2 mg/kg, remifentanil 1 g/kg, and rocuronium bromide 0.6 mg/kg. Anesthesia was maintained by target-controlled infusion of propofol + remifentanil to keep the bispectral index of electroencephalogram at 40–60.

After anesthesia induction, the control group was subjected to ultrasound-guided brachial plexus block: patients were placed in supine after general anesthesia, and the muscular sulcus plexus was located under ultrasound-guided position. A puncture needle (22G 80 mm) was used to puncture the intra-plane, and 0.375% ropivacaine 20 mL (150 mg) was injected into the anterolateral and posterolateral brachial plexus.

After anesthesia induction, the research group performed serratus anterior plane block under ultrasound guidance: the patient was placed in supine after general anesthesia, and the latissimus dorsi muscle between the midaxillary line and the posterior axillary line was located under ultrasound guidance. The needle was inserted into the plane from top to bottom until the serratus anterior surface, and 0.375% ropivacaine 20 mL was slowly injected.

Arthroscopic shoulder surgery was performed 20 min after the block operation in both groups. After surgery, patients were installed with an intravenous controlled analgesia pump (PCIA), which was formulated as follows: 100 *μ*g sufentanil + 5 mg tropisetron hydrochloride + 98 mL normal saline, background infusion of 2 mL/h, single additional dose of 0.5 mL, locking time of 15 min. The standard process of clinical trial report of this study is shown in Figure 1.

### 2.3. Evaluation Indexes

The visual analogue scale (VAS) was used to score the analgesic effect of patients at 6, 12, 24, 48, and 72 h after surgery [9]: The total score is 0∼10, 0 is painless and 10 is severe pain. The lower the score, the lighter the pain, the better the analgesic effect. The patient can move the cursor on the scale to evaluate the pain.

The intraoperative dosage of propofol and remifentanil, the effective pressing times of analgesic pump within 48 h after operation, the first pressing time of analgesic pump, and the total amount of sufentanil were recorded.

The levels of pain mediators and oxidative stress factors were compared between the two groups at 3 days after surgery: 5 mL of fasting venous blood was taken from patients, and serum was taken after centrifugation. ①Pain mediators: serum levels of calcitonin gene-related peptide (CGRP) and neuropeptide Y (NPY) were measured by enzyme-linked immunosorbent assay. ②Oxidative stress factors: serum malondialdehyde (MDA) levels and superoxide dismutase (SOD) enzyme activity were detected by the reflex immunoprecipitation method. All operations were carried out in strict accordance with the kit instructions.

Adverse analgesic reactions such as nausea and vomiting, skin itching, and dizziness were recorded within 72 h after operation.

### 2.4. Statistical Methods

Data were processed by SPSS 22.0 software, VAS scores and other measurement materials were expressed as mean ± standard deviation ($\bar{x}$ ± *s*), and intergroup comparison was performed by independent sample *T-*tests. The incidence of adverse reactions was expressed as %, and x^2^ tests were applied. Bilateral inspection: inspection level is *α* = 0.05, with *P* < 0.05; the difference was statistically significant.

## 3. Results

### 3.1. Comparison of VAS Scores between the Two Groups at Different Time Points

At 6, 12, 48, and 72 h after surgery, there was no significant difference in VAS scores between the two groups (*P* > 0.05); 24 h after surgery, the VAS score of the study group was significantly lower than that of the control group (*P* < 0.05) (Table 2).

### 3.2. Comparison of Intraoperative Anesthetic Dosage between the Two Groups

The intraoperative doses of propofol and remifentanil in the study group were significantly lower than those in the control group (*P* < 0.05) (Table 3).

### 3.3. Comparison of Postoperative Analgesic Drug Use between the Two Groups

The effective pressing times of analgesic pump and the total amount of sufentanil in the study group were significantly lower than those in the control group within 48 hours after operation, and the first pressing time of analgesic pump was significantly longer than that in the control group (*P* < 0.05; Table 4).

### 3.4. Comparison of the Levels of Pain Mediators and Oxidative Stress Factors between the Two Groups

Before surgery, there were no significant differences in the levels of CGRP, NPY, and MDA and SOD enzyme activity between the two groups (*P* > 0.05). After surgery, the levels of pain mediators CGRP and NPY in the study group were lower than those in the control group (*P* < 0.05); the level of oxidative stress factor MDA in the study group was lower than that of the control group, and SOD was higher than that of the control group (*P* < 0.05; Table 5).

### 3.5. Comparison of the Occurrence of Adverse Reactions between the Two Groups

In the study group, nausea and vomiting occurred in 2 cases and dizziness occurred in 1 case, and the incidence of adverse reactions was 6.38% (3/47). In the control group, there were 3 cases of nausea and vomiting, 1 case of pruritus, and 1 case of vertigo, and the incidence of adverse reactions was 10.64% (5/47). There was no significant difference in the incidence of adverse reactions between the two groups (*x*^2^ = 0.547, *P* > 0.05).

## 4. Discussion

Arthroscopic shoulder surgery has become one of the main ways to treat shoulder diseases with less trauma and faster recovery than traditional open surgery [10, 11]. The anatomical structure of shoulder joint is complex, and arthroscopic shoulder surgery is prone to severe pain, especially in the early postoperative stage [12]. Postoperative pain causes the body to produce a large number of pain mediators and causes oxidative stress. Effective control of postoperative pain is very important to improve patient comfort and clinical treatment effect.

The ideal analgesic method should have the advantages of simple operation, complete analgesia, less use of anesthetic drugs, lasting effect, and fewer complications [13, 14]. Secondly, the long-term movement block of the affected limb will affect the postoperative rehabilitation exercise, and because the local anesthetic is easy to spread to the phrenic nerve on the surface of the anterior scalene muscle, the risk of phrenic nerve block is high. Ultrasound-guided intermuscular sulcus brachial plexus block is a common way of anesthesia for arthroscopic shoulder surgery, which has the advantages of simplicity and easy operation. However, this method needs to be injected into the anterior upper and posterior lateral of the brachial plexus, and the posterior lateral branch also receives the impulse of sensory branch nerve from the thoracic nerve. In arthroscopic surgery, this area is the surgical entrance, so it is easy to increase patients' pain [15, 16]. As a new local anesthesia method, ultrasound-guided serratus anterior plane block is mainly used to inject local anesthesia between latissimus dorsi muscle and serratus anterior muscle to block the T2–T9 sensory plane of the lateral cutaneous branch of the intercostal nerve and achieve analgesic effect on the anterolateral chest wall. Therefore, this study compared the analgesic effect, anesthetic drug use, and adverse reactions of ultrasound-guided brachial plexus block and ultrasound-guided anterior serratus plane block to comprehensively explore the analgesic efficacy and adverse reactions of ultrasound-guided anterior serratus plane block in arthroscopic shoulder surgery from subjective and biochemical objective indexes and to provide reference for the selection of anesthesia operation methods and reduce patients' pain.

The VAS score is used to evaluate the pain degree of patients and can reflect the analgesic effect of patients. This study found that the VAS score of the study group was significantly lower than that of the control group 24 h after surgery. The amount of propofol and remifentanil in the study group was significantly lower than that in the control group, the number of effective pressing of analgesic pump and the total amount of sufentanil used within 48 h after operation were significantly lower than that in the control group, and the time of first pressing of analgesic pump was significantly longer than that in the control group. Ultrasonic-guided serratus anterior plane block can provide longer and more complete analgesia for patients undergoing arthroscopic shoulder surgery. The anterior plane is a fascia space, located on the inner side of scapula and the posterior side of latissimus dorsi. Under the guidance of ultrasound, 0.375% ropivacaine 20 mL was injected between latissimus dorsi and serratus anterior, and the range of sensory block was T2–T9 (covering the anterior, posterior, and lateral chest walls), so as to achieve the analgesic effect. The brachial plexus nerve block can avoid touching the anterior upper and posterolateral brachial plexus and reduce the pain of patients. Wang et al. [16] also found that 0.375% ropivacaine 20 mL used for serratus anterior plane block can significantly reduce the postoperative VAS pain score of breast cancer patients, enhance the analgesic effect, and reduce the use of opioids. Takimoto et al. [17] proved that serratus anterior plane block can produce analgesic effect by blocking the lateral cutaneous branch.

Arthroscopic shoulder surgery causes trauma to patients due to a wide range of involvement in the operation process, and patients usually have varying degrees of pain after surgery, which causes the body to produce a large number of pain mediators and trigger oxidative stress response [18, 19]. CGRP is a neuropeptide that can sensitize pain and reduce pain threshold. NPY is a common pain mediator, which can mediate pain signal transmission. MDA is a decomposition product of oxidative reaction, and its content can reflect the degree of tissue damage caused by oxidative stress. SOD is an antioxidant enzyme that catalyzes the reduction reaction [20]. The results of this study showed that, after surgery, the levels of pain mediators CGRP and NPY in the study group were lower than those in the control group, the level of oxidative stress factor level of MDA was lower than that in the control group, and the activity of SOD was higher than that in the control group. These results indicate that ultrasound-guided serratus anterior block can effectively inhibit postoperative pain and oxidative stress in patients undergoing arthroscopic shoulder surgery. This may be due to the fact that this anesthesia method can avoid touching the anterior upper and posterolateral brachial plexus with brachial nerve block in the intermuscular groove, which reduces the pain of patients and leads to a higher comfort level and less stress response. In addition, there was no significant difference in the occurrence of analgesic adverse reactions such as nausea and vomiting, skin itching, and dizziness between the two groups. However, it can be seen that this anesthesia method has high safety about the actual adverse reactions. Liu et al. [21] applied ultrasound-guided serratus anterior muscle block to patients undergoing thoracotomy and found that this anesthesia method did not lead to blockage-related complications with good safety.

## 5. Conclusion

Ultrasonic-guided serratus anterior plane block has a good anesthetic effect in arthroscopic shoulder surgery and lasting effect time, can significantly reduce the amount of opioids, enhance postoperative analgesia, and effectively inhibit postoperative pain and oxidative stress response of patients, with good safety.

## Figures and Tables

**Figure 1:** Flow diagram of trial.

**Table 1:** Comparison of general data between the two groups ($\bar{x}$ ± *s*).

Group	Count	Cases gender [*n* (%)]		ASA [*n* (%)]		Age (years)	Operation time (min)
		Male	Female	Grade I	Grade II		
The study group	47	28(59.57)	19(40.43)	37(78.72)	10(21.28)	48.26 ± 10.14	69.38 ± 19.62
The control group	47	30(63.83)	17(36.17)	39(82.98)	8(17.02)	49.12 ± 9.85	71.67 ± 21.85
*χ* ^2^/*t*		0.180		0.275		0.417	0.535
*P*		0.671		0.600		0.678	0.594

**Table 2:** Comparison of VAS scores between the two groups at different time points ($\bar{x}$ ± *s*, scores).

Group	Case	After 6 h	After 12 h	After 24 h	After 48 h	After 72 h
The study group	47	1.85 ± 0.59	2.69 ± 0.75	2.86 ± 0.83	2.17 ± 0.65	1.47 ± 0.43
The control group	47	1.91 ± 0.62	2.85 ± 0.81	3.24 ± 0.96	2.38 ± 0.71	1.54 ± 0.48
*T*		0.481	0.994	2.053	1.496	0.745
*P*		0.632	0.323	0.043	0.138	0.458

**Table 3:** Comparison of intraoperative anesthetic dosage between the two groups ($\bar{x}$ ± *s*).

Group	Case	Propofol (mg)	Remifentanil (*μ*g)
The study group	47	41.95 ± 14.47	26.71 ± 8.15
The control group	47	50.14 ± 16.95	31.24 ± 9.86
*T*		2.519	2.428
*P*		0.013	0.017

**Table 4:** Comparison of postoperative analgesic use between the two groups ($\bar{x}$ ± *s*).

Group	Case	Effective pressing times of analgesic pump within 48 h after surgery (times)	Time of the first pressing of the analgesic pump (h)	Total sufentanil usage (*μ*g)
The study group	47	4.15 ± 1.24	12.15 ± 2.45	105.17 ± 8.95
The control group	47	4.81 ± 1.57	10.96 ± 2.13	110.03 ± 9.64
*t/χ* ^2^		2.262	2.513	2.633
*P*		0.026	0.014	0.013

**Table 5:** Comparison of the levels of pain mediators and oxidative stress factors between the two groups ($\bar{x}$ ± *s*）.

Groups	Case	CGRP (*μ*g/L)		NPY (*μ*g/L)		MDA (*μ*mol/L)		SOD (U/L)	
		Preoperative	Postoperative	Preoperative	Postoperative	Preoperative	Postoperative	Preoperative	Postoperative
The study group	47	104.75 ± 16.83	198.74 ± 32.69^a^	78.92 ± 9.15	137.64 ± 20.85^a^	5.19 ± 1.07	11.72 ± 2.38^a^	67.85 ± 9.13	47.62 ± 8.37^a^
The control group	47	102.98 ± 15.49	221.37 ± 35.71^a^	79.54 ± 8.96	150.17 ± 23.59^a^	5.24 ± 1.12	13.52 ± 3.16^a^	68.39 ± 8.95	43.75 ± 8.24^a^
*T*		0.531	3.205	0.332	2.728	0.221	2.426	0.290	2.259
*P*		0.597	0.002	0.741	0.008	0.825	0.017	0.773	0.026

Note. Compared with this group before operation, ^a^*P* < 0.05.

## Data Availability

The simulation experiment data used to support the findings of this study are available from the corresponding author upon request.
